# Qualitative and quantitative determination of chemical constituents in Jinbei oral liquid, a modern Chinese medicine for coronavirus disease 2019, by ultra-performance liquid chromatography coupled with mass spectrometry

This article has been retracted.

**DOI:** 10.3389/fchem.2023.1079288

**Published:** 2023-02-07

**Authors:** Aijun Zhang, Qingcui Xu, Juanjuan Jiang, Zimo Zhao, Liangzong Zhang, Kai Tao, Guiyun Cao, Jinghua Zhang, Lin Ding, Zhaoqing Meng, Wenyao Dong, Chunxia Wang

**Affiliations:** ^1^ Traditional Chinese Medicine Research Institute, Shandong Hongjitang Pharmaceutical Group Co., Ltd., Jinan, China; ^2^ Faculty of Veterinary and Agricultural Sciences, University of Melbourne, Parkvile, VIC, Australia; ^3^ Institute of Optical Physics and Engineering Technology, Qilu Zhongke, Jinan, China; ^4^ The first Clinical Medical College of Shandong University of Traditional Chinese Medicine, Jinan, China; ^5^ Yinan County People’s Hospital, Linyi, China

**Keywords:** Jinbei oral liquid, quadrupole time-of-flight mass spectrometry, qualitative analysis, triple quadrupole mass spectrometry, quantitative analysis

## Abstract

**Introduction:** Traditional Chinese medicine (TCM) has the advantages of syndrome differentiation and rapid determination of etiology, and many TCM prescriptions have been applied to the clinical treatment of coronavirus disease 2019 (COVID-19). Among them, Jinbei Oral Liquid (Jb.L) has also shown an obvious curative effect in the clinic, but the related material basic research is relatively limited.

**Methods:** Therefore, in this process, a systematic data acquisition and mining strategy was established using ultra-high- performance liquid chromatography coupled with quadruple time-of-flight mass spectrometry (UPLC-Q-TOF-MS).

**Results and Discussion:** With the optimized conditions, a total of 118 peaks were tentatively characterized, including 43 flavonoids, 26 phenylpropanoids, 14 glycosides, 9 phthalides, 8 alkaloids and others. To determine the content of relevant pharmacological ingredients, we firstly exploited the ultra-performance liquid chromatography method coupled with triple-quadrupole tandem mass spectrometry (UPLC-QqQ-MS/MS) method for simultaneous detection of 31 active ingredients within 17 min, and the validation of methodology showed that this method has good precision and accuracy. Moreover, analyzing the pharmacology of 31 individual of the medicinal material preliminarily confirmed the efficacy of Jb.L and laid a foundation for an in-depth study of network pharmacology.

## 1 Introduction

In December 2019, many cases of viral pneumonia were found in Wuhan City, Hubei Province. By February 2020, more than 20,000 cases of coronavirus disease 2019 (COVID-19) were confirmed nationwide, and 425 patients had died. For this outbreak, it is difficult for western medicine to carry out targeted treatment without identifying the pathogen, but traditional Chinese medicine (TCM) can quickly determine the cause through syndrome differentiation and treatment (Zeng et al., 2020).

COVID-19 belongs to the category of “epidemic disease” in TCM, and its pathological changes first appear in the interstitial lung (Yang and Fan, 2021). The main symptoms are fever, dry cough, and fatigue. In severe cases, lung consolidation may occur (Miao et al., 2020; Xiong, 2020; Zhan et al., 2020). In view of these symptoms, many prescriptions were applied, such as Jinhua Qinggan granules, Shufeng Jiedu capsules, Jingfang granules, and Jinbei oral liquid (Jb. L), and showed an obvious curative effect in the clinic. Among them, Jb. L was listed in the Chinese Medicine Diagnosis and Treatment Plan of novel coronavirus pneumonia in Shandong Province (Second Edition) in February 2020, and our subsequent clinical data analysis showed that the effect of Jb. L combined with chemical drugs was better than the single chemical therapy group (Li et al., 2021). Jb. L is composed of *Astragali radix*, *Codonopsis radix*, *Angelica sinensis*, *Glehniae radix*, *Scutellariae radix*, *Fritillariae cirrhosae bulbus*, *Chuanxiong rhizoma*, *Salvia miltiorrhiza radix*, *Pinelliae rhizoma praeparatum cumalumine*, *Lonicerae japonicae flos*, *Forsythiae fructus*, *and Glycyrrhizae radix*. It has the effect of replenishing qi and nourishing yin, expelling blood stasis, and removing phlegm.

Although TCM prescriptions have a certain theoretical and clinical application basis, the material basis of compound TCM prescriptions is complex, and the action mechanism is diverse, which brings considerable difficulty to the basic material research into the efficacy of TCM. In recent years, hyphenated techniques have been powerful tools for rapid online qualitative analysis of unknown compounds in complex matrices, especially ultra-performance liquid chromatography coupled with quadrupole time-of-flight tandem mass spectrometry (UPLC-Q-TOF-MS), which benefits due to its high resolution and sensitivity. These methods have been proven to be efficient and highly sensitive tools for the rapid analysis of TCM preparations (Gao et al., 2014; Zhang et al., 2017a; Li et al., 2018; Wang et al., 2018; Sun et al., 2021). In addition, UPLC coupled with triple quadrupole mass spectrometry (UPLC-QqQ-MS/MS) can be well applied to quantitative analysis of multiple chemical components of TCM through the multiple reaction monitoring (MRM) mode, which has great significance in the modernization of TCM (Wu et al., 2019; Liu et al., 2020; Zheng et al., 2021).

Studying the material basis of the efficacy of TCM is the prerequisite to solving the principle of the effective action of TCM, and the determination of the effective components of TCM is the primary task. Therefore, in this experiment, the chemical composition of Jb. L was qualitatively determined by UPLC-Q-TOF-MS/MS, and the main functional components were quantitatively analyzed by UPLC-MS/MS. This is the first report on the systematic analysis of the chemical components of Jb. L, which provides the basis for quality control and an in-depth study of its pharmacodynamics.

## 2 Materials and methods

### 2.1 Instruments and reagents

An Agilent 1290 UPLC system was coupled with an Agilent 6530C Q-TOF-MS/MS (Agilent Technologies, USA); A Waters ACQUITYTM I-Class UPLC (Waters Technologies, USA) was coupled with a SCIEX Triple Quad 5,500 (AB SCIEX, USA); an XS105 analytical balance was purchased from METTLER TOLEDO (Shanghai, China); a KQ-800VSM Bench ultrasonic cleaner was purchased from Kunshan Ultrasonic Instrument Co., Ltd. (Jiangsu, China); LC-MS-grade acetonitrile was purchased from Merck KGaA (Darmstadt, Germany); HPLC-grade formic acid was purchased from Kermel (Tianjin, China); ultra-pure water was purchased from Watsons (Guangzhou, China).

A total of 31 reference standards (adenosine, guanosine, chlorogenic acid, loganin, caffeic acid, schaffetaside, rutin, forsythoside A, ferulic acid, sibemine, fritillin B, isochlorogenic acid A/B/C, quercitrin, rosmarinic acid, salvianolic acid B, liquiritin, lindenaza, baicalin, genistein, forsythin, liquiritigenin, mullein isoflavones, bergamot esters, baicalein, formononetin, glycyrrhizic acid, glycyrrhetinic acid, wogonin, and ligustilide) were purchased from the National Institutes for Food and Drug Control, Jiangsu Yongjian Pharmaceutical Technology, Ltd., and Shandong WoDeSen Bioscience Technology, Ltd. The purities of all the reference standards were over 96.0%. Samples of Jb. L were produced by Shandong Hongjitang Pharmaceutical Group, Ltd.

### 2.2 Preparation of reference standards and sample solutions

Individual reference standards were prepared by accurately weighing the required amounts and dissolving the in LC-MS-grade methanol. Samples were stored at 4 °C before being analyzed.

The Jb. L sample (20 mL) was extracted ultrasonically for 30 min once with 60 mL of methanol. After it was cooled to room temperature, the weight was supplemented. The sample was filtered through a 0.22 μm nylon membrane filter before being analyzed.

### 2.3 Method of qualitative analysis by UPLC-Q-TOF-MS/MS

The research was performed on a Poroshell 120 SB-C18 column (2.1 mm *150 mm, 2.7 μm) at a flow rate of 0.2 mL/min, and the injection volume was 2 μL. To obtain good chromatographic separation and appropriate ionization, the UPLC-Q-TOF-MS/MS conditions were optimized systemically. Similarly, the column, temperature, and elution profile were optimized for LC. Different sheath gases and collision energies were investigated for MS. The mobile phase was composed of 0.1% (v/v) formic acid (A) and acetonitrile (B) with gradient elution, and the elution program was as follows: 0–2.7 min, 4% B; 2.7–6.6 min, 4%–7% B; 6.6–20.6 min, 7%–14% B; 20.6–30.7 min, 14%–19% B; 30.7–43.9 min, 19%–30% B; 43.9–54.3 min, 30%–50% B; 54.3–64 min, 50%–70% B; 64–75 min, 70%–80% B.

Mass spectrometric conditions were as follows: both positive and negative electrospray ionization (ESI) modes were applied to this analysis. The capillary voltage was 3.5 kV (negative ion mode) and 4.0 kV (positive ion mode), and the collision energy range of the secondary mass spectrum was 20–60 eV. MS scan and auto MS/MS modes were adopted, the scanning range of mass spectrometry was 100–1,200 Da, and the data acquisition was centroid mode.

### 2.4 Method of quantitative analysis by UPLC-QqQ-MS/MS

The analysis was performed on an ACQUITY UPLC BEH C18 column (2.1 mm *100 mm, 1.7 μm). The mobile phase was 0.1% formic acid (A) and acetonitrile (B) with gradient elution (0–1.0 min,10% B; 1.0–3.0 min, 10%–20% B; 3.0–5.0 min, 20%–30% B; 5.0–7.0 min, 30%–40% B; 7.0–9.0 min, 40%–55% B; 9.0–11.0 min, 55%–70% B; 11.0–14.0 min, 70%–80% B; 14–15 min, 80%–85% B; 15.0–16.1 min, 85%–10% B; 16.1–17 min, 10% B); the flow rate was 0.3 mL/min. Mass spectrometric conditions were as follows: ionization of analytes was carried out using positive/negative mode electrospray ionization (ESI) with the multiple reaction monitoring (MRM) mode. The ion source spray voltage was 4500 V, the curtain gas was 20.0 psi, the ion source gas was 50 psi, the entrance potential was ±10 V, and the collision cell exit potential was ±5.5 V. The MS analysis parameters of 31 detected compounds are shown in Table 1, and the extracted ion chromatograms of each component are shown in Supporting Information Figure S2. The data acquisition and processing software was MultiQuant 3.0.2 Workstation.

**TABLE 1:** MS analysis parameters of 31 detected compounds.

No.	Compound	Retention time/min	Precursor ion m/z	Production m/z	Collision energy/eV	Declustering potential/v	Ionization mode	No.	Compound	Retention time/min	Precursor ion m/z	Production m/z	Collision energy/eV	Declustering potential/v	Ionization mode
1	Imperialine	4.54	430.9	412.4/138.2	43/61	70/70	ESI+	17	4,5-Dicaffeoylquinic acid	498	515.1	352.9/173.0	27/34	112/115	EST-
2	Peiminine	4.55	430.1	412.7/3963	58/74	72/72	ESI+	18	Caffeic acid	298	179.1	134.9/107.1	27/31	89/71	EST-
3	Liquiritin	5.54	419.0	137.0/147.2	54/45	119/143	ESI+	19	Chlorogenic acid	238	353.1	190.9/178.9	20/21	60,94	BSI-
	Glycyrrhizic acid	837	823.3	453.4/647.3	37/19	139/129	ESI+	20	Luteoloside	5.66	447.1	285.0/327.0	37/34	62/121	BSI-
5	Liquiritigenin	6.04	255.4	119.0/91.0	30/32	67/68	ESI-	21	Rutin	4.01	609.1	299.7/270.9	49/69	134/79	BSI-
6	180-Glycyrrhetinic acid	838	471.1	189.1/317.2	47/42	58/93	ESI+	22	Forsythin	598	557.3	309.1/185.0	36/3	140/118	BSI+
7	Baicalein	7.75	271.0	123.0/103.1	42.141	138/137	EST+	23	Forsythoside A	4.18	623.2	160.9/179.0	48/48	140/140	PSI-
8	Wogonin	9.02	285.5	269.9/179.0	43/46	31/38	EST+	24	Ligustilide	10.71	191.5	91.1/117.1	38/27	141/141	ESI+
9	Rosmarinic acid	5.12	359.0	161.0/178.8	49/50	57/77	BSI-	25	Ralik acid	430	193.0	133.9/177.8	23/18	92/123	PSI-
10	Baicalin	5.67	445.7	269.8/175.0	29/15	77177	BSI-	26	Bergapten	7.45	217.5	202.1/174.1	29/38	85/119	ESI+
11	Schaftoside	3.49	563.2	443.0/353.0	38/46	140/127	BSI-	27	Calycosin	6.28	283.0	268.0/210.9	37/45	92/92	EST-
12	Formononetin	8.17	267.6	252.9/132.0	27/40	120/120	BSI-	28	Genistin	5.70	433.2	271.2/415.3	28/42	91/42	ESI+
13	Salvianolic acid B	5.46	717.8	320.9/518.9	45/25	22/21	BSI-	29	Adenosine	0.82	268.1	135.9/118.8	25/62	71/78	ESI+
14	Loganin	2.68	413.1	219.0/251.2	33/29	109/109	ESD-	30	Guanosine	1.02	284.2	152.3/135.2	16/49	51/49	ESI+
15	3,5-Dicaffeoylquinic acid	4.69	515.1	353.0/191.1	21/47	86/71	BSI-	31	Quercitrin	4.69	447.1	254.9/299.8	53/35	52/53	BSI-
16	3,4-Dicaffeoylquinic acid	4.57	515.2	353.1/172.9	38/27	116/112	BSI-								

## 3 Results

We herein report the qualitative and quantitative analysis of the chemical constituents of Jb. L using both UPLC-Q-TOF-MS/MS and UPLC-QqQ-MS/MS. The research diagram is shown in Figure 1.

**FIGURE 1:** Research strategy for identifying the components of Jinbei oral liquid See Supplementary Figure S1.

### 3.1 Identification of chemical compositions by UPLC-Q-TOF-MS/MS

The total ion chromatograms (TIC) of Jb. L samples were obtained under chromatographic and mass spectrometry conditions described in Section 2.3. These chromatograms are shown in Figure 2. First, according to the chromatographic peak information, the molecular formula was generated by the Compound Identification function in Agilent Qualitative Workflows B.08.00 software. The compounds contained in Jb. L were preliminarily identified by comparison with the relevant literature on the chemical constituents of 12 TCMs (Zhang and Ye, 2009; Song et al., 2014; Su et al., 2015; Xia et al., 2016; Zhang et al., 2017b; Huang et al., 2018; Jiang et al., 2020; Luo et al., 2020; Wang and Su, 2020; Yao et al., 2020; Zhang et al., 2020; Zhao and Xia, 2020). Second, the corresponding fragment ions of the compound were obtained by secondary mass spectrometry of collision-induced dissociation (CID). As a result, 118 compounds were detected and tentatively identified in Jb. L by comparing the retention time and mass spectrometry and retrieving the reference literature. These compounds included 43 flavonoids, 26 phenylpropanoids, 14 glycosides, 9 phthalides, 8 alkaloids, and others. The quality deviation was controlled within 15 ppm. The structures of these compounds are summarized in Figure 3. Information on the t_R_ (min), molecular formula, theory mass (*m/z*), observed mass (*m/z*), mass error (in ppm), fragment ions, and category is summarized in Supporting Information Table S1. Among them, 31 components, such as chlorogenic acid, caffeic acid, salvianolic acid B, baicalin, glycyrrhizic acid, cryptotanshinone, imperialine, forsythin, calycosin, schaftoside, rutin, and so on, were compared with the corresponding reference standards.

**FIGURE 2:** UPLC-Q-TOF-MS total ion chromatogram of Jinbei oral liquid in negative **(A)** and positive **(B)** ion mode See Supplementary Figure S2.

**FIGURE 3:** Potential chemical structures investigated in Jinbei oral liquid See Supplementary Figure S3.

#### 3.1.1 Flavonoids

Flavonoids are secondary plant metabolites with various pharmacological effects. They are a series of compounds with 2-phenylchromone as the basic parent nucleus and mainly have anti-inflammatory, antioxidant, cardiovascular protection, and other effects. For example, rutin can significantly inhibit the activity of cardiac inflammation and can play a protective role against cardiac inflammation (Dai et al., 2013; Alara et al., 2018). It is abundant in Chinese herbal medicinal plants, such as *Astragalus*, *Scutellaria*, *Glycyrrhiza*, and *Forsythia*. In this study, the 45 identified flavonoids can be divided into four classes (flavonoids, dihydroflavonoids, isoflavones, and pterocarpoids). The compounds include schaftoside (12), hesperidin (13), liquiritin (14), and liquiritigenin-7-O-D-apiosyl-4’-O-D-glucoside (15), and luteoloside (17), baicalin (29), calycosin (36), wogonoside (38), rutin (69), hyperoside (70), quercitrin (73), pratensein 7-O-*β*-D-glucopyranoside (78), genistin (84), methylnissolin-3-O-glucoside (90), baicalein (100), isoastragaloside IV (101), formononetin (106), and so on. The mass spectra information is shown in Supporting Information Table S1.

##### 3.1.1.1 Flavonoids

The identification process of flavonoids is illustrated by taking schaftoside and kumatakenin as examples. Schaftoside produced ion *m/z* 563.1400 [M-H]^-^ in negative source mode. In its secondary mass spectrometry, molecules of H_2_O (18 Da) and Glc (162 Da) were removed to produce a fragment ion fragment *m/z* 383.0770, followed by either the removal of a CH_2_O (30 Da) molecule to produce fragment ion *m/z* 353.0665 or the removal of a C_4_H_8_O_4_ (120 Da) molecule to produce fragment ion *m/z* 443.0960. The possible fragmentation pathway (FP) is shown in Figure 4A. In the positive ion mode, kumatakenin exhibited an [M + H]^+^ ion at *m/z* 315.0866 (1.27 ppm, C_17_H_14_O_6_), then neutral elimination of a CH_3_ (15 Da) residue produced the ion at *m/z* 299.0571 ([M + H-15]^-^, C_16_H_11_O_6_). The ion at *m/z* 243.0642 ([M + H-56]^-^, C_14_H_11_O_4_) came from the neutral elimination of a C_2_O_2_ residue. In addition, C_1_-C_3_ of the A-ring directly underwent RDA cleavage to produce fragment ion *m/z* 167.0317 ([M + H-C_9_H_7_O_2_]^-^, C_8_H_7_O_4_). The possible FP is shown in Figure 4B.

**FIGURE 4:** **(A)** The FP of schaftoside in negative ion mode. **(B)** The FP of kumatakenin in positive ion mode. **(C)** Mass spectrometric fragmentation of dihydroflavones. **(D)** The FP of liquiritin in negative ion mode. **(E)** The FP of formononetin in positive ion mode. **(F)** The FP of calycosin-7-O-glucoside in positive ion mode. **(G)** The FP of methylnissolin-3-O-glucoside in positive ion mode.

##### 3.1.1.2 Dihydroflavonoids

In the positive source mode, the parent C-ring of dihydroflavonoids generally undergoes a ring-opening rupture with break sites at the C2-*O* and C3-C4 bonds, generating ions retained at the A-ring end (RDA cleavage). In the negative source mode, break sites at the C2-*O* and C4-C10 bonds also occur at the same time, generating ions with charge retained at the A-ring end, sometimes with the loss of the B-ring, as shown in Figure 4C. The identification process of dihydroflavonoids is illustrated taking liquiritin as an example. Liquiritin underwent glycosidic bond breakage in both positive and negative ion modes, and one molecule of the glucose group was removed to obtain a fragment ion with *m/z* 255.0662 [M-H-Glc]^-^. Then, RDA cleavage occurred in the C-ring to produce fragment ion *m/z* 135.0085. The FP is shown in Figure 4D.

##### 3.1.1.3 Isoflavones

For isoflavones, in positive ion mode, the primary mass spectra were obtained with [M + H]^+^ peaks, and the other fragments were formed by the absence of neutral units such as CO, CH_3_, and CHO or the occurrence of RDA cleavage. The identification process of isoflavones is illustrated by the example of formononetin and calycosin-7-*O*-glucoside. In the positive source mode, formononetin produced excimer ion *m/z* 269.0807 [M + H]^+^. Fragment ions *m/z* 137.0238 and *m/z* 133.0643 were generated after RDA cleavage, and then neutral elimination of CHO (29 Da) and CH_3_ (15 Da) produced the ions at *m/z* 108.0211 and *m/z* 118.0409, respectively. Formononetin may also remove one molecule of CH_3_ (15 Da) and then remove one H atom to obtain fragment ions of *m/z* 253.0469. The possible cleavage pathway is shown in Figure 4E. The fragment ion m/z 285.0766 was found in the positive ion mode because the oxyglycoside bond was prone to break and one molecule of the glycosyl group was removed, to obtain the fragment ion *m/z* 285.0766, and then one molecule of CH_3_ (15 Da) or CH_4_O (32 Da) was also lost to produce the fragment ion *m/z* 270.0532 or *m/z* 253.0481. The *m/z* 270.0532 fragment ion underwent RDA cleavage to yield a fragment ion of *m/z* 137.0232, and its possible FP is shown in Figure 4F.

##### 3.1.1.4 Pterocarpoids

Pterocarpins are second only to isoflavones in the isoflavone family. The basic skeleton is a tetracyclic system synthesized by the 4-position and 2′-position of isoflavones through ether bond rings. Pterocarpin has two asymmetric carbon atoms, C-6a and C-11a. The identification process of pterocarpoids is illustrated by taking methylnissolin-3-*O*-glucoside as an example. In the positive ion mode, methylnissolin-3-*O*-glucoside produced an [M + H]^+^ ion at *m/z* 463.1601 (0.65 ppm, C_23_H_26_O_10_); the fragment ion *m/z* 301.1086 showed an ionized peak corresponding to the ion *m/z* 463.1601 losing a glucose group. Meanwhile, it showed 162 Da more than compound 89, indicating more glycosyl (Glc, 162 Da) than medicarpin. Finally, the fragment ion at *m/z* 167.0711 was generated after removing substituents (C_8_H_6_O_2_, 144 Da), and its possible FP is shown in Figure 4G.

Obviously, for flavonoids, the fragmentation of MS is mainly the cleavage of sugar residues or small molecules and the cleavage of RDA in the ring.

#### 3.1.2 Phenylpropanol

Phenylpropanol is a naturally occurring compound composed of a benzene ring and three straight-chain carbon groups (C6-C3 groups) and can be divided into phenylpropionic acids, coumarins, and lignans.

##### 3.1.2.1 Phenylpropionic acids and derivatives

The structure of phenylpropionic acid is characterized by a C6-C3 structure and aromatic carboxylic acid substituted by a phenolic hydroxyl group. Danshensu (1), 5-*O*-caffeoylquinic acid (3), 1-O-caffeoylquinic acid (7), chlorogenic acid (9), cryptochlorogenic acid (10), caffeic acid (11), lithospermic acid (19), 3,4-dicaffeoylquinic acid (20), 3,5-dicaffeoylquinic acid (21), rosmarinic acid (24), 4,5-dicaffeoylquinic acid (25), salvianolic acid B (31), salvianolic acid E (33), and salvianolic acid A (35) were the main phenylpropionic acids in Jb. L. They can be divided into three types according to the different substituents of compounds: caffeoyl substituents, salvianolic acids, and other organic acids (Zhang et al., 2006; Lin et al., 2017; Cao et al., 2021). For example, compounds 20, 21, and 25 are three typical caffeoyl-substituted phenolic acids that produced similar precursor ions at *m/z* 515.1194 and fragment ions at *m/z* 353.0873 [M-H-Caff]^-^ in negative ion mode, and *m/z* 191.0551 [M-H-2Caff]^-^, *m/z* 179.0350 [M-H-Caff-C_7_H_10_O_5_]^-^, *m/z* 173.0450 [M-H-2Caff-H_2_O]^-^, and *m/z* 135.0462 [M-H-Caff-C_7_H_10_O_5_-CO_2_]^-^ the identification of the last four fragment ions is based on literature and mass spectrometry analysis. Taking 4,5-dicaffeoylquinic acid as an example, the main FP of caffeoyl-substituted phenolic acids is summarized in Figure 5A. Salvianolic acid compounds are the main water-soluble compounds in *Salvia miltiorrhiza*, among which the two components with the highest content, salvianolic acid A and B, have the strongest activity. Salvianolic acids A and B are compounds with danshensu as the parent nucleus. In the negative ion mode, salvianolic acid B exhibited an [M-H]^-^ ion at *m/z* 717.1459 (0.84 ppm, C_36_H_30_O_16_), then split in the CID mode and lost danshensu to produce fragment ions at *m/z* 519.0928, *m/z* 339.0505, and *m/z* 321.0402 corresponding to [M-H-C_9_H_10_O_5_]^−^, [M-H-C_9_H_10_O_5_-C_9_H_8_O_4_]^−^ and [M-H-2C_9_H_10_O_5_]^−^, respectively. The secondary mass spectra are shown in Figure 5B. The FP was inferred as shown in Figure 5C. Rosmarinic acid is used as an example of other organic acids. Rosmarinic acid is a diploid synthesized by caffeic acid and danshensu condensation, and the most unstable one is the intermediate ester bond. As shown in Figure 5D, fragment ions *m/z* 161.0240 and *m/z* 197.0449 were formed when the bond was broken, and fragment ion *m/z* 179.0346 was formed when the charge was broken by the b bond. The final structure was the same whether the charge was on the caffeic acid or danshensu. The inferred cleavage law was also confirmed according to the secondary mass spectra of rosmarinic acid and its standard (Figure 5E). Other types of acids tend to lose stable small molecules or free radicals. For example, lithospermic acid has a phenylpropionic acid unit, which is triploid, and the unstable part of the structure is lactone and carboxyl groups on the benzodihydrofuran ring. The FP is shown in Figure 5F.

**FIGURE 5:** **(A)** MS/MS spectrogram of salvianolic acid B in negative ion mode. **(B)** The FP of salvianolic acid B in negative ion mode. **(C)** MS/MS spectrogram of rosmarinic acid in negative ion mode (A-sample, B-reference standard). **(D)** The FP of rosmarinic acid in negative ion mode. **(E)** The FP of lithospermic acid in negative ion mode. **(F)** The FP of terpineol in negative ion mode. **(G)** The FP of7-hydroxycoumarin in positive ion mode.

##### 3.1.2.2 Lignans

Lignans are defined as a class of natural products formed by the connection of two structures with a phenylpropane skeleton by the β,β′ or 8,8-carbons, mainly including forsythin (85), sylvatesmin (86), and terpineol (95). Taking terpineol as an example, the molecular fragment peak mainly comes from the benzene ring and the cyclic alkyl group. In positive ion mode, terpineol is produced an [M + H]^+^ ion at *m/z* 359.1489 (1.39 ppm, C_20_H_22_O_6_), then neutral elimination of H_2_O (18 Da), 2 OCH_2_ (60Da), and C_6_H_4_ (76 Da) to produce the ion at *m/z* 205.0842. Similarly, after the loss of a small molecule, fragment ions at *m/z* 151.0375 and *m/z* 137.0605 were also obtained. The possible FP is shown in Figure 5G.

##### 3.1.2.3 Coumarin

Coumarin is a lactone compound synthesized by intramolecular dehydration cyclization of cis-o-hydroxycinnamic acid. It has the basic core nucleus of benzopyranone and has been found in *Angelica sinensis radix* and *Glycyrrhiza radix*. Variants include liquiritigenin (31), 7-hydroxy coumarin (51), hydroxymethyl couman (57), scopoletin (58), fraxidin (62), bergapten (96), 8-methoxypsoralen (107), phellopterin (110), and so on. In the positive source mode, the excimer ion was at *m/z* 163.0391 [M + H]^+^, and a molecule of CO (28 Da) was removed successively to form characteristic fragments at *m/z* 135.0449 [M + H-CO]^+^, *m/z* 107.0500 [M + H-2CO]^+^, and *m/z* 79.0545 [M + H-3CO]^+^, respectively. The FP is shown in Figure 5H.

#### 3.1.3 Glycosides

Glycosides, also known as glycoplasts, are compounds formed by connecting the terminal carbon atoms of sugars or sugar derivatives with another kind of non-sugar substance (called aglycone, ligand or aglycone). Fourteen glycosides were identified in Jb. L, including phenylethanol glycosides such as forsythoside A (16), forsythoside E (52), salidroside (53), and desrhamnosyl isoacteoside (64); nucleosides, such as adenosine (46) and guanosine (47); saponins, such as astragaloside *II* (42), astragaloside *VI* (93), astragaloside *IV* (101), licoricesaponin *G*2 (105), glycyrrhizic acid (108), 18*β*-glycyrrhetinic acid (109), and so on. Generally, it is difficult to observe molecular ions in these compounds, and sometimes only molecular ions with extremely low abundance can appear. However, the fragment ions produced by continuous dehydration of molecular ions or dehydration after deglycosylation, as well as fragment ions from the aglycone and glycosyl parts, can be clearly seen.

The glycyrrhizic acid in triterpene saponins is used as an example. There is a double glucuronic acid (-GluA) in its structure. In the positive ion mode, the *m/z* 647.3776 was a fragment that lost a molecule of dehydrated glucuronic acid. Then, the charge was on the 11-position carbonyl of glycyrrhetinic acid, and the dehydrated diglucuronic acid was lost to obtain *m/z* 471.3464 [M + H-2GluA]^+^. There were hydrogen atoms on both sides of the sugar and aglycone of the 3-position glycosidic bond, so, in addition to *m/z* 471.3464, one molecule of H_2_O can also be lost to form *m/z* 453.3357 [M + H-2GluA-H_2_O]^+^. Its secondary mass spectrum is shown in Figure 6A, and the possible FP is shown in Figure 6B.

**FIGURE 6:** **(A)** MS/MS spectrogram of glycyrrhizic acid in positive ion mode; **(B)** the FP of glycyrrhizic acid in positive ion mode; **(C)** the FP of astragaloside IV in positive ion mode; **(D)** MS/MS spectrogram of forsythoside A in negative ion mode; **(E)** the FP of forsythoside A in negative ion mode.

The structure of astragaloside IV contains a glucose group (-Glc) and a xylose group (-Xyl). In the positive ion mode, the fragment ion *m/z* 491.3694 [M + H-Glc-Xyl]^+^ was obtained after removing the sugar group, then neutral elimination of H_2_O (18 Da) produced *m/z* 455.3518 [M + H-Glc-Xyl-2H_2_O]^+^ and *m/z* 437.3395 [M + H-Glc-Xyl-3 H_2_O]^+^. After the removal of 3 H_2_O, the C-C bond between the two five-membered rings breaks to form fragment ion *m/z* 143.1067 [M + H-Glc-Xyl-3H_2_O-C_22_H_30_]^+^ with a spiroketal structure, and its possible FP is shown in Figure 6C.

Taking forsythoside A with high content in *Forsythia suspensa* as an example: in negative ion mode, the [M-H]^-^ *m/z* 623.1965 ion produced fragment ions representing *m/z* 461.1683, *m/z* 443.1536, and *m/z* 179.0346 due to the successive losses of C_9_H_6_O_3_ (162 Da), H_2_O (18 Da), and C_13_H_12_O_6_ (264 Da), respectively. The secondary mass spectrum is shown in Figure 6D, and the possible FP is shown in Figure 6E.

#### 3.1.4 Phthalide

Phenylphthalide, also known as o-hydroxymethylbenzoic acid lactone, is structurally characterized as a bicyclic fusion of *γ*-lactone (A-ring) and benzene (B-ring), a lactone formed by the loss of one molecule of H_2_O from *γ*-hydroxy carboxylic acid. It has antibacterial, analgesic, and anti-inflammatory biological activities, with significant therapeutic effects in calming asthma, lowering blood pressure, and improving the immune system (Zhang et al., 2017c). *Angelica sinensis* and *Chuanxiong rhizoma* are rich in phenanthrenes. In this study, a total of nine phenanthrenes were identified, including senkyunolide *J/I/F/H/G/A* (65, 77, 79, 80, 103, 113) and 3-butylphthalide (102), *E*-ligustilide (114), and *Z*-ligustilide (116). In the positive ion mode, the senkyunolide *J/I/H/G* excimer ion was dominated by [M + Na]^+^, and the senkyunolide F/A excimer ion was dominated by [M + H]^+^ followed by the loss of small molecules H_2_O, CO, CO_2_ to produce fragment ions. Compounds 104, 116, and 118 have the same excimer ion at *m/z* 191 [M + H]^+^ and have the same fragment ion *m/z* 173 [M + H-H_2_O]^+^, presumably with a similar cleavage pattern (Lin et al., 1998). Among them, *E*-ligustilide and *Z*-ligustilide are cis-trans isomers with significantly different retention times according to the relevant literature, and the peak of *E*-ligustilide is earlier. *E*-ligustilide is used as an example to illustrate the identification process of phenylpeptides: it yielded an ion at *m/z* 191.1065 [M + H]^+^ in the positive ion mode, and the molecular formula was estimated to be C_12_H_14_O_2_ by mass spectrometry software. After removing small molecules of H_2_O (18 Da) and CO (28 Da), respectively, fragment ions were produced at *m/z* 173.0961, *m/z* 163.1138, and *m/z* 145.1015, and the possible FP is shown in Figure 7.

**FIGURE 7:** The FP of E-ligustilide in positive ion mode.

#### 3.1.5 Alkaloids

Alkaloids are a class of nitrogenous organic compounds originating from the biological world (mainly the plant world), most of which have a more complex ring structure with nitrogen atoms bound within the ring. Alkaloids have protective effects on the cardiovascular system. For example, the alkaloid fraction in the Chinese herbal medicine maidenhair has pharmacological effects such as lowering blood pressure, slowing heart rate, and anti-tumor, in addition to its cough suppressing, asthma calming, and expectorant effects. Eight alkaloids were identified in this study, corresponding to compounds such as phenylalanine (49), tryptophan (50), mussel methycin (61), imperialine (67), perlolyrine (72), peimine (74), peiminine (76), and 1-acetyl-carboline (104). Imperialine is used as an example to illustrate the identification process of alkaloids. The *m/z* displayed in positive ion mode was 430.3320 [M + H]^+^. In its secondary mass spectrum, the excimer ion lost one molecule of H_2_O (18 Da) to yield *m/z* 412.3214 fragment ion, followed by a retro Diels–Alder (RDA) reaction that produced a fragment ion at *m/z* 138.1266 ([M + H-C_18_H_26_O_2_]^+^, C_19_H_16_N), and its possible FP is shown in Figure 8.

**FIGURE 8:** The FP of imperialine in positive ion mode.

#### 3.1.6 Other compounds

Many other substances were also found in Jb. L, such as tanshinones, including tanshinone I (118), cryptotanshinone (117), and dihydrotanshinone I (115), iridoid terpenoids, including sweroside (56), loganin (57), and secoxyloganin (60), and triterpenes, including ursolic acid (98) (Wang et al., 2020). Cryptotanshinone is used as an example. In ESI^+^ mode, the excimer ion was *m/z* 297.1490 [M + H]^+^(1.68 ppm,C_19_H_20_O_3_) with fragments at *m/z* 279.1375 [M + H-18]^+^ and *m/z* 251.1411 [M + H-46]^+^, corresponding to [M + H-H_2_O]^+^ and [M + H-H_2_O-CO]^+^, respectively. Cryptotanshinone might also direct shed C_2_H_5_(29 Da) to form a fragment ion *m/z* 268.1120. The possible FP is shown in Figure 9A. Taking sweroside as an example, the *m/z* displayed in the ESI^+^ mode was 359.1340 ([M + H]^+^). After CID cleavage, the fragment ion *m/z* 197.0809 corresponding to excimer ion losing a glucose group, then neutral elimination of H_2_O/CO/C_4_H_4_ residue produced the ions at *m/z* 179.0691 ([M + H-Glc-18]^+^), *m/z* 151.0747 ([M + H-Glc-18-28]^+^), and *m/z* 127.0392 ([M + H-Glc-18-52]^+^). The possible FP is shown in Figure 9B.

**FIGURE 9:** **(A)** The FP of cryptotanshinone in positive ion mode; **(B)** the FP of sweroside in positive ion mode.

### 3.2 Quantitative analysis by UPLC-QqQ-MS/MS

#### 3.2.1 Preparation of reference standards

Adenosine, guanosine, chlorogenic acid, loganin, caffeic acid, schaffetaside, rutin, forsythoside A, ferulic acid, sibemine, fritillin B, isochlorogenic acid A/B/C, quercitrin, rosmarinic acid, salvianolic acid B, liquiritin, lindenaza, baicalin, genistein, forsythin, liquiritigenin, mullein isoflavones, bergamot esters, baicalein, formononetin, glycyrrhizic acid, glycyrrhetinic acid, wogonin, and ligustilide reference substances were accurately weighed in appropriate amounts, dissolved in methanol and diluted to make a mass concentration of 100 ppm of the reference stock solution. A 0.1 mL aliquot of each of the above-mentioned reference substances was added to a 10 mL volumetric flask. Methanol was added to dilute to scale, and the flask was shaken well to obtain the No. 1 mixed reference substance solution. The No. 1 mixed reference solution was diluted 2, 4, 5, 10, and 20 times to prepare mixed reference solutions Nos. 2–6.

#### 3.2.2 Methodological investigation of quantitative detection methods

##### 3.2.2.1 Investigation of extraction methods

Five samples of Jb. L were selected at random and fully mixed. A 10 mL aliquot of the mixed solution was precisely measured and dissolved into 30 mL of 50% (V/V) methanol-water solution and shaken.

The samples were treated separately by the following methods: ultrasonic extraction for 30 min (250 W, frequency 40 kHz); reflux for 30 min. Then, the sample was allowed to cool to room temperature. The sample was weighed, and the weight loss reduction was made up with the 50% (v/v) methanol-water solution. The sample was shaken well and filtered through a 0.22 μm microporous filter. The early filtrate was abandoned, and the subsequent filtrate was taken as the sample solution. The total ion chromatograms of different extraction methods are shown in Figure 10. It can be seen from the figure that ultrasonic and reflux extraction have no significant effect on the chromatographic peak response of the components in the sample. In view of the stable baseline of the chromatographic peaks produced by ultrasonic extraction, ultrasonic extraction was determined to be more appropriate.

**FIGURE 10:** Total ion chromatograms of Jinbei oral liquid by different extraction methods. **(A)** Ultrasonic; **(B)** reflux See Supplementary Data Sheet 2.

##### 3.2.2.2 Investigation of extraction solvents

A 10 mL sample of Jb. L was extracted with 30% methanol, 50% methanol, and 80% methanol as extraction solvents, respectively. The sample solution was prepared according to the ultrasonic extraction method described in Section 3.2.2.1, and the sample was injected for analysis. The TIC diagrams of the samples with different extraction solvents are shown in Figure 11. The chromatographic peak response of the components extracted by 50% methanol was high, and the baseline was relatively stable, so 50% methanol was selected as the extraction solvent.

**FIGURE 11:** Total ion chromatograms of Jinbei oral liquid by different extraction solvents. **(A)** 30% methanol; **(B)** 50% methanol; **(C)** 80% methanol See Supplementary Data Sheet 3.

##### 3.2.2.3 Investigation of extraction time

A 10 mL sample of Jb. L was precisely measured, and 50% methanol was used as the extraction solvent. The sample was ultrasonically extracted for different durations (20, 30, 40 min) to prepare the test solution, which was then injected and analyzed. The TIC of the sample under different extraction times is shown in Figure 12. Considering the response value of the chromatographic peak and the stability of the baseline, the extraction time was selected as 30 min.

**FIGURE 12:** Total ion chromatograms of Jinbei oral liquid by different extraction times. **(A)** 20 min; **(B)** 30 min; **(C)** 40 min See Supplementary Data Sheet 4.

##### 3.2.2.4 Confirmation of sample preparation method

According to the above investigation results, it was determined that the sample solution preparation method was as follows: 10 mL of Jb. L was accurately measured and transferred to a stoppered conical flask; 30 mL of 50% methanol was accurately added. The sample was precisely weighed and subjected to ultrasonic extraction for 30 min. After cooling to room temperature, the weight was made up, the solution was filtered, and the filtrate was used for analysis.

##### 3.2.2.5 Stability test

The sample solution of Jb. L was injected after 0, 2, 6, 12, and 24 h. The results (Supporting Information Figure S3) showed that the RSD values of 31 compounds were in the range of 1.62%–4.70%, which indicated that the content of the test solution was stable within 24 h, and it was appropriate to inject samples for analysis within this time range.

##### 3.2.2.6 Repeatability test

The same batch of Jb. L was weighed in parallel with six portions, and the sample solution was prepared according to the method described in Section 3.2.2.4. The contents of 31 compounds were analyzed and calculated (Supporting Information Figure S3). The RSD was in the range of 2.49%–5.59%, indicating that the method has good repeatability.

##### 3.2.2.7 Precision test

The 31 compounds in Jb. L were divided into three groups. The mixed reference substance *A* containing peiminine, bergapten, 18β-glycyrrhetinic acid, imperialine, quercetin, genistin, and formononetin was prepared with a concentration of 250 ng/mL. Mixed reference solution *B* containing calycosin, liquiritigenin, loganin, schaftoside, rutin, wogonin, luteoloside, ferulic acid, and guanosine was prepared with a concentration of 2.5 μg/mL. Mixed reference solution C containing baicalein, ligustilide, adenosine, rosmarinic acid, forsythin, caffeic acid, isochlorogenic acid A/B/C, liquiritin, glycyrrhizic acid, chlorogenic acid, baicalin, salvianolic acid B, and forsythoside A was prepared with a concentration of 10 μg/mL. Three 5-mL samples were taken from the same batch of Jb. L. A 1 mL sample of the reference solutions A, B, and C was added to each, respectively. The results showed that the recovery rate was in the range of 91.2%–109.4%, indicating that the accuracy of the method was good.

##### 3.2.2.8 Durability test

The durability was investigated in two aspects: column temperature and chromatographic column. The setting of column temperature was varied by ±2 °C (33 °C and 37 °C), and different batches of the same brand of column material were selected for the chromatographic column. The results showed that the durability of the system meets the requirements, and the RSD of the measured concentration was less than 4.5%.

##### 3.2.2.9 Linear relationship and sample determination

A 2 μL sample of each of the six reference solutions No. 1 to No. 6 mentioned in Section 3.2.1 was injected. Taking the peak area as the ordinate (y) and the mass concentration (μg·L^−1^) as the abscissa (x), a standard curve was drawn to obtain the regression equation and correlation coefficient (r) of each component. The result is shown in Table 2 and indicates that all components have a good linear relationship and high sensitivity.

**TABLE 2:** Calibration curves and determination of 31 compounds detected in Jinbei oral liquid.

No.	Compound	Linear equation	Correlation coefficient	Content/(μg/mL)	No.	Compound	Linear equation	Correlation coefficient	Content/(μg/mL)
1	Imperialine	y = 5,827.2x-521.13	R.^2^ = 0.9988	0.43	1	4,5-Dicaffeoylquinic acid	y = 2673.8x −19959	li.^2^ = 0.9963	57.98
2	Peiminine	y = 26236x+78109	R.^2^ = 0.9998	0.03	I s	Caffeic acid	y = 3779.5x+ 13427	P.^2^ = 0.9993	30.83
3	Liquiritin	y = 342.8x +7708.6	W = 0.9933	43.46	19	Chloroganc acid	y = 2507.6x + 46783	R' = 0.9944	75.14
4	Glygrrhizic acid	y = 2401.41 E+26052	R.^2^ = 0.9947	63.93	20	Luteoloside	y = 3634.3x + 75209	R' = 0.9971	752
5	Liquiritigenin	y = 2958x+50925	R.^2^ = 0.9987	*336*	21	Rutin	y = 2903.8x+ 13218	12.^2^ = 0.9998	4.74
6	1813-Glycyrrhetinic acid	y = 997.13x+1698.9	R.^2^ = 0.9922	0.18	22	Forsythin	y = 109.47x + 1888.1	12.^2^ = 0.9972	25.76
7	Baicalein	y = 2080.1x - 28289	R.^2^ = 0.9972	11.98	23	Fcasythoside A	y = 599.56x + 9257.4	R' = 0.9950	776.70
8	Wogonin	y = 9225.5x+ 107086	R.^2^ = 0.9988	554	24	Ligustilide	y = 520.38x - 4362.7	W^.^ = 0.9988	12.96
9	Rosmarinic acid	y = 534.67x + 5,438.6	R.^2^ = 0.9975	24.29	25	Rosmarinic acid	y = 711.29x + 10180	R' = 0.9990	820
10	Baicalin	y = 129.68x + 2059.1	R.^2^ = 0.9908	13L61	26	Bergapten	y = 6139.2x - 52792	R' = 0.9983	0.11
11	Schaftosicie	y = 517.03x + 2832.6	R.^2^ = 0.9971	4.69	27	Calycosin	y = 4076.2x + 79611	R' = 0.9964	115
12	Formononetin	y = 410.96x + 3150.6	R.^2^ = 0.9986	1.08	28	Genistin	y = 4831.5x - 77873	R' = 0.9965	0.91
13	Salvianolic acid B	y = 99.444x + 1925.3	R.^2^ = 0.9965	17338	29	Adenosine	y = 5,762.2x - 100.47	R' = 0.9979	14.40
14	Loganin	y = 66.5x + 11992	R.^2^ = 0.9978	4.25	30	Guanosine	y = 4195.4x - 339.23	R.: = 0.9995	9.62
15	3,5-Dicaffeoyiquinic acid	y = 1624.1x + 24541	R.^2^ = 0.9900	37.94	31	Quercitrin	y = 375.88x + 1527.1	R.: = 1.0000	0.90
16	3,4-Dicaffeoyiquinic acid	y = 1704.8x + 669.65	R.^2^ = 0.9966	55.19					

Three batches of Jb. L samples were prepared according to the method described in Section 3.2.2.4 and analyzed within 24 h, and the contents of adenosine, guanosine, chlorogenic acid, and 31 other components in the samples were calculated as shown in Table 2. The results show that the components with the highest concentrations were forsythoside A, which has bacteriostatic and anti-inflammatory effects; flavonoids with antioxidant effects, such as calycosin, baicalin, liquiritin, rutin; salvianolic acid B, chlorogenic acid, rosmarinic acid, and other organic acids with anti-inflammatory and antibacterial effects; and adenosine, guanosine, and other nucleosides with immune regulation functions. Alkaloids with antitussive, expectorant, and anti-inflammatory effects, such as imperialine and peiminine, were found with the next-highest concentrations.

## 4 Discussion

The material basis for prevention and treatment within TCM is an organic whole composed of multiple components, which is a prerequisite for elucidating the active substances, pharmacological action, mechanism, and clinical efficacy of TCM. Therefore, in the process of research and development for new TCM drugs, it is necessary to strengthen basic research, discover clinical characteristics and comparative advantages, focus on clinical positioning, and improve clinical efficacy.

In this study, UPLC-Q-TOF-MS was used to qualitatively analyze various chemical components in Jb. L, and a total of 118 compounds were detected and tentatively identified, including 43 flavonoids, 26 phenylpropanoids, 14 glycosides, 9 phthalides, 8 alkaloids, and others. Among them, 31 compounds were analyzed and compared with reference materials by mass spectrometry. Other components were analyzed by comparing the mass spectrometry and retrieving the reference literature. It may also be necessary to further analyze and verify with reference materials. We developed a UPLC-QqQ-MS/MS method for the simultaneous determination of 31 effective constituents in Jb. L. Formononetin, calycosin, and genistin from *Astragali radix* are flavonoids and important antioxidant active substances. Ligustilide, bergapten, and ferulic acid are the main active ingredients in *Angelica sinensis* and *Chuanxiong rhizoma* and have many physiological activities such as spasmolysis, asthma relief, sedation and analgesia, and myocardial protection. Baicalin, baicalein, and luteoloside are the main active substances in *Scutellariae radix* and have antiviral effects *in vivo* and *in vitro*. Liquiritin, liquiritigenin, glycyrrhizic acid, 18*β*-glycyrrhetinic acid, and schaftoside are the main active ingredients in *Glycyrrhizae radix*. From the perspective of network pharmacology reported in the literature, liquiritin can inhibit the expression of IL-17 inflammatory factors and has an anti-inflammatory effect. Liquiritigenin can regulate the Th1 immune response, and glycyrrhizic acid can inhibit the proliferation of fibroblasts, induce cell cycle arrest and promote cell apoptosis. 18β-Glycyrrhetinic acid can inhibit the production of the coronavirus by interfering with the early stage of virus replication. Schaftoside has the effects of protecting the liver, resisting inflammation, clearing heat, and eliminating dampness. Salvianolic acid B and rosmarinic acid are derived from *Salvia miltiorrhiza radix*. Salvianolic acid B can inhibit inflammatory cell infiltration, alveolar structure destruction, and collagen deposition in animal experiments. Rosmarinic acid has strong anti-inflammatory, antibacterial, and antiviral activities. Forsythin, forsythoside A, and quercitrin are from *Forsythiae fructus* and have good anti-inflammatory effects. The main antiviral components of *Lonicerae japonicae flos* are flavonoids and organic acids, such as chlorogenic acid, isochlorogenic acid A/B/C, caffeic acid, and rutin, which are quantitatively analyzed in this study, and they are the main markers of *Lonicerae japonicae flos*’s heat-clearing and detoxification effects. Imperialine and peiminine are derived from *Fritillariae cirrhosae bulbus* and have the effects of relieving cough, eliminating phlegm, and blocking the production of pro-inflammatory mediators. Adenosine and guanosine are alkaloids commonly contained in twelve TCMs and have the effect of regulating immunity.

The above ingredients confirmed the material basis of Jb. L’s pharmacological activities of invigorating qi, nourishing yin, removing blood stasis, and resolving phlegm. However, we can only infer from the pharmacology reported in the literature, and further research is needed.

In this paper, 118 compounds from Jb. L were identified and analyzed, and a quantitative analysis method for 31 active ingredients was established. Moreover, the verification results of the methodology prove that the quantitative analysis method has good specificity, high sensitivity, and short analysis time, providing a powerful means for the rapid and accurate analysis of the complex system of a Chinese patent medicine preparation. We expect that this strategy may provide a good basis for future research on the metabolomics and network pharmacology of Jb. L and other TCM prescriptions.

## Data Availability

The original contributions presented in the study are included in the article/Supplementary Material; further inquiries can be directed to the corresponding author.
